The article "Diagnostic dilemma in a patient with history of medullary thyroid carcinoma and abnormal serum liver enzymes; a case report with six years follow up" was published in 2023. Journal: BMC Endocr Disord.

# Diagnostic dilemma in a patient with history of medullary thyroid carcinoma and abnormal serum liver enzymes; a case report with six years follow up

**DOI:** 10.1186/s12902-023-01439-7

**Published:** 2023-08-30

**Authors:** Fatemeh Rahmani, Maryam Tohidi, Farid Azmoudeh-Ardalan, Amir Sadeghi, Farzad Hadaegh

**Affiliations:** 1 Prevention of Metabolic Disorders Research Center, Research Institute for Endocrine Sciences, Shahid Beheshti University of Medical Sciences, No. 24, Yamen Street, Velenjak, Tehran, Iran; 2 Department of Pathology, Cancer Institute, Imam Khomeini Hospital Complex, Tehran University of Medical Sciences, Tehran, Iran; 3 Gastroenterology and Liver Diseases Research Center, Shahid Beheshti University of Medical Sciences, Tehran, Iran

**Keywords:** Case report, Medullary thyroid carcinoma, Histopathology, Neuroendocrine tumor, Primary biliary cholangitis

## Abstract

**Background:**

Medullary thyroid carcinoma (MTC) is a neuroendocrine tumor that originates from parafollicular C-cells. Calcitonin (Ctn) and carcinoembryonic antigen (CEA) are useful biomarkers for monitoring MTC cases.

**Case presentation:**

Here, we describe a 48-year-old woman, who presented in 2014 with bilateral thyroid nodules. Report of fine needle aspiration was suspicious for MTC; initial laboratory evaluation showed serum Ctn level of 1567 pg/mL. After excluding type 2 multiple endocrine neoplasia syndrome clinically, total thyroidectomy and neck lymph node dissection were performed. The final histopathological diagnosis was right lobe MTC with neither vascular invasion nor lymph node involvement. On regular follow-up visits, Ctn and CEA levels have been undetectable, and repeated cervical ultrasonographic exams were unremarkable from 2014 to 2021. As liver enzymes became elevated in 2016, the patient was further evaluated by a gastroenterologist. Abdominopelvic ultrasonography revealed a coarse echo pattern of the liver parenchyma with normal bile ducts. A liver fibroscan showed a low fibrosis score (7kPa). The patient was recommended to use ursodeoxycholic acid. According to the progressive rise of liver enzymes with a cholestatic pattern in October 2020, a liver biopsy was performed that showed tiny nests of neuroendocrine-like cells with a background of primary biliary cholangitis (PBC). Immunohistochemical stainings were positive for chromogranin A (CgA), and synaptophysin and negative for Ctn, CEA, and thyroglobulin. Further imaging investigations did not reveal any site of a neuroendocrine tumor in the body. Considering normal physical exam, imaging findings, as well as normal serum levels of Ctn, CEA, CgA, and procalcitonin, the patient was managed as a PBC.

The article "Diagnostic dilemma in a patient with history of medullary thyroid carcinoma and abnormal serum liver enzymes; a case report with six years follow up" was published in 2023. Journal: BMC Endocr Disord.

**Conclusion:**

In follow-up of a patient with MTC, we reported progressively increased liver enzymes with a cholestatic pattern. Liver biopsy revealed nests of neuroendocrine-like cells with a background of PBC, the findings that might suggest acquiring neuroendocrine phenotype by proliferating cholangiocytes.

## Background

Medullary thyroid carcinoma (MTC) is a rare differentiated neuroendocrine tumor (NET), that originates from thyroid parafollicular C-cells, with an occurrence rate of 2–5% among all thyroid cancers [1]. C-cells of the thyroid gland produce several hormones and biogenic amines [2]. Calcitonin (Ctn) and carcinoembryonic antigen (CEA) are well-recognized biomarkers secreted from neoplastic C-cells in well-differentiated MTC. Considering the high sensitivity and specificity of these biomarkers, they are applied for monitoring the remission versus disease progression in individuals with MTC [2–4].

According to the revised American thyroid association (ATA) guideline, thyroid nodules suspected for or diagnosed as MTC in cytological or histopathological examinations, respectively, should be managed with neck ultrasound examination, determinations of serum Ctn and CEA levels, and DNA analysis for the rearranged during Transfection (RET) germline mutation [5]. In sporadic MTC, after total thyroidectomy and central neck lymph node dissection, follow-up by physical examination, neck ultrasonography, serum Ctn, and CEA levels are recommended [5]. Although, metastatic cases of MTC with normal serum levels of biomarkers were reported [2, 6], generally undetectable serum Ctn and CEA levels, in combination with a negative residual tumor on imaging examinations, exclude the presence of metastatic MTC [7].

In our case, a MTC with clinical and paraclinical remission, gradually rising liver enzymes with the presence of neuroendocrine-like cells in the liver biopsy could be explained by changes in the phenotype of cholangiocytes to neuroendocrine-like cells.

## Case presentation

A 48-year-old woman, with no personal or family history of thyroid malignancy, was consulted for thyroid nodules in November 2014. Physical examination revealed multiple nodules in both thyroid lobes, without compression effects on adjacent organs. Ultrasonography of the neck documented one hypoechoic nodule 44 × 28 mm with microcalcification in the right lobe and two 14 × 8 mm and 9 × 6 mm isoechoic nodules in the left lobe with no neck lymphadenopathy. Fine needle aspiration cytology of the right lobe nodule was reported as suspicious for MTC and serum Ctn level was 1567 pg/mL (reference value: < 10 pg/mL). The patient was clinically and biochemically euthyroid. Her blood pressure was 110/70 mmHg. She did not complain of paroxysmal hypertension, palpitation, or sweating; also, she did not have personal or family history of renal stone or hypercalcemia. Laboratory tests including serum calcium, parathyroid hormone, and 24-h urine collection for vanillylmandelic acid, norepinephrine, and epinephrine were unremarkable (Table 1). The patient was scheduled for total thyroidectomy and bilateral cervical lymph node dissection in November 2014. Histopathological examination confirmed the diagnosis of right lobe MTC without vascular invasion, extracapsular extension, lymph node involvement, or C-cell hyperplasia. Immunohistochemical (IHC) stainings were positive for Ctn, synaptophysin, chromogranin A (CgA), and negative for thyroglobulin (Tg). RET mutation in the patient’s peripheral blood lymphocytes was positive in exon 11, codon 691, and exon 15, codon 904. Two months after thyroidectomy, serum Ctn and CEA levels were 1.3 pg/mL (reference value: < 10 pg/mL) and 4.9 ng/mL (reference value: < 2.5 ng/mL), respectively; with mildly elevated liver enzymes i.e., aspartate aminotransferase: 44 IU/L, alanine aminotransferase: 38 IU/L, and alkaline phosphatase (ALP): 380 IU/L. Since the calcium-loaded calcitonin test was not available at that time and considering the immediate post-operative significant decrement of serum calcitonin level, this test was not performed. On regular follow-up visits, serum Ctn and CEA levels were consistently below the upper limit of reference ranges from 2014 to 2021 (Fig. 1), and repeated cervical ultrasonography did not show abnormal findings. According to gradually raised liver enzymes with a cholestatic pattern (Fig. 2), the patient was referred to a gastroenterologist for evaluation of liver function in 2016. Abdominopelvic ultrasonography revealed a coarse echo pattern of the liver with normal internal and external bile ducts. Liver fibroScan showeda low fibrosis score (7kPa). Anti-mitochondrial antibody was 1.2 units (reference value: < 1.5 units), and other immunological tests and hepatitis serology panels were normal. Treatment with ursodeoxycholic acid 300 mg daily was initiated and the patient followed clinically and biochemically. Since liver enzymes especially ALP and gamma glutamyl transferase (GGT) gradually elevated in 2020, a liver biopsy was performed. The histopathological examination of the liver biopsy, reported by two experienced pathologists, showed tiny nests of neuroendocrine-like cells, severe portal lymphoplasma cell infiltration, some piecemeal necrosis, mild bile duct proliferation, focal parenchymal destruction of interlobular bile ducts by granulomatous reaction, and fibrous expansion of portal tracts with occasional p-p bridges (Fig. 3). IHC staining showed diffuse mild to moderate positivity for synaptophysin. IHC staining for CgA was positive in 80% of cells with moderate intensity (Fig. 4). Negative results were reported for Ctn, CEA, and Tg. The proliferation marker of Ki67 was positive in 2–3% of the neuroendocrine-like cells. Histopathologic findings and IHC stainings were compatible with the presence of neuroendocrine-like cells in a background of primary biliary cholangitis (PBC). Results of upper and lower gastrointestinal endoscopies, whole body bone scan with TC^99^ and ^68^Ga-Dotatate positron emission tomography (PET)-CT scan were unremarkable. Abdominal computed tomography (CT) showed few periportal and portocaval lymph nodes (up to 10 × 14 mm). Endoscopic ultrasound evaluation only suggested a few hilar and peripancreatic lymph nodes. Subsequent FNA of hilar lymph node was negative for NET or any other malignancy, and IHC stainings were negative for cytokeratin, synaptophysin, Ctn, and CgA. Serum CgA and procalcitonin levels were reported 43 ng/mL (reference value: < 100 ng/mL) and 0.1 ng/mL (reference value: < 0.15 ng/mL), respectively. Hence, according to negative biochemical and radiological evidence for primary or secondary hepatic NETs, as well as the presence of obstructive liver pathology, the final diagnosis of anti-mitochondrial autoantibodies (AMA)-negative PBC was made and the patient was managed with glucocorticoid.

The article "Diagnostic dilemma in a patient with history of medullary thyroid carcinoma and abnormal serum liver enzymes; a case report with six years follow up" was published in 2023. Journal: BMC Endocr Disord.

**Table 1:** Laboratory tests on the first admission in October 2014

Test	Patient value	Reference range
White blood cell	7700//mm^3^	4500–11,000/mm^3^
Hemoglobin	14 g/dL	13.5–17.5 g/dL
Platelets	178,000 /mm^3^	150,000–450,000/mm^3^
Erythrocyte sedimentation rate	14 mm/hour	0–20 mm/hour
Blood urea nitrogen	14 mg/dL	8–20 mg/dL
Creatinine	0.9 mg/dL	0.5–1.5 mg/dL
Alanine aminotransferase	27 IU/L	5–40 IU/L
Aspartate aminotransferase	34 IU/L	5–40 IU/L
Alkaline phosphatase	243 U/L	44–147 U/L
Thyroid stimulating hormone	1.65mIU/L	0.5–5 mIU/L
Total thyroxine	9.4 mcg/dL	5–12 mcg/dL
Calcium	9.4 mg/dL	8.6–10.6 mg/dL
Phosphate	3.9 mg/dL	2.5–4.5 mg/dL
Parathyroid hormone	18 pg/mL	10–55 pg/mL
Calcitonin	1547 pg/mL	< 10 pg/mL
24 h urine epinephrine	5 mcg/24 h	0.5–20 mcg/24 h
24 h urine norepinephrine	24 mcg/24 h	15–80 mcg/24 h
24 h urine vanillylmandelic acid	7.3 mcg/24 h	< 13.5 mcg/24h

**Fig. 1:** Trend of basal serum Ctn and CEA levels from 2014 to 2021. Ctn: calcitonin, CEA: carcinoembryonic antigen

**Fig. 2:** Trend of serum liver enzymes levels. ALT: Alanine aminotransferase, AST: Aspartate aminotransferase, ALP: alkaline phosphatase

**Fig. 3:** Histopathologic sections of the liver biopsy (×100 and × 400 magnifications): **A** and **B**, Liver tissue with cholestatic pattern of injury and bile duct damage (H&E stain); **C** and **D**, Fibrous expansion of portal tract with occasional p-p bridges (Trichrome stain); **E** and **F** Nests of neuroendocrine-like cells (H&E stain)

**Fig. 4:** Immunohistochemistry (IHC) stained sections of the liver biopsy (×100 and × 400 magnifications): **A** and **B**. IHC staining for Chromogranin **A**; **C** and **D**, IHC staining for synaptophysin

The article "Diagnostic dilemma in a patient with history of medullary thyroid carcinoma and abnormal serum liver enzymes; a case report with six years follow up" was published in 2023. Journal: BMC Endocr Disord.

## Discussion and conclusions

Here, we reported a case of MTC with high serum Ctn level and no neck lymph node involvement at presentation. After total thyroidectomy, the patient had been in a complete biochemical and clinical remission, with undetectable serum biomarkers and normal neck sonography through 6 years. During follow-up, a gradual rising of liver enzymes with a cholestatic pattern was seen. Histopathological evaluation of liver biopsy revealed tiny nests of neuroendocrine-like cells in a background predominantly with a cholestatic pattern, in favor of PBC, although imaging findings indicated no evidence of metastasis.

Three potential scenarios could be proposed for our case. Considering the patient’s history of MTC, the most probable explanation for the presence of nests of neuroendocrine-like cells in the liver biopsy was late metastatic MTC to the liver with low serum Ctn level. MTC, an uncommon and aggressive thyroid cancer, could occur sporadically or hereditary as a component of type 2 multiple endocrine neoplasia syndrome [6]. Regarding the sequence of the coding region of RET proto-oncogene mutation in this case that was not in moderate or high-risk categories, as well as considering the occurrence of somatic RET mutation in 50% of sporadic MTCs [5], we considered this patient as a sporadic case of MTC and followed her with repeated cervical neck ultrasonographic exams and serum Ctn and CEA levels in approximately 6–12 month intervals. C-cells of the thyroid gland secrete several hormones and biogenic amines [5], Ctn and CEA are two useful tumor markers secreted from these cells in MTC. Although these biomarkers could be increased in different conditions [5], their monitoring is helpful in postoperative follow-up and determining the prognosis of individuals with MTC [7]. In rare cases of metastatic MTC, serum Ctn and CEA levels could be normal or undetectable. Several reasons have been advocated to explain this medical dilemma. The hook effect is one of the possible explanations; however, in our case, we did not recheck the Ctn level in serially diluted samples. Some authors hypothesize dedifferentiation as a leading cause of the inability of a tumor to produce Ctn [2]. Studies reported various behavior of MTC regardless of the initial stage and the presence or absence of distant metastasis ranging from prolonged indolent course to highly aggressive one [8]. Recently, Park et al. evaluate the clinical characteristics and long-term oncologic outcomes of 46 MTC cases with distant metastasis. According to this study, the cancer-specific- survival for patients with MTC and isolated liver metastasis were reported to be 100.0% at one, three, five, and 10 years, respectively. However, the corresponding values for patients with multi-organ metastasis were 84.6%, 53.8%, 46.2%, and 30.8%, respectively [9] In our patient, diagnostic evaluation for metastatic MTC including whole body scan, abdominopelvic CT, ^68^ Ga-Dotatate PET-CT, and EUS could not detect any focus of malignancy.

The article "Diagnostic dilemma in a patient with history of medullary thyroid carcinoma and abnormal serum liver enzymes; a case report with six years follow up" was published in 2023. Journal: BMC Endocr Disord.

Metastatic liver NET of unknown origin versus primary hepatic NET (PHNET) might be considered as the second scenario. The liver is the most common site for metastatic NET of the gastrointestinal tract and pancreas in the majority of cases [10, 11], but PHNET is a rare disease with an incidence rate of 0.17% [12]. PHNETs are slightly predominant in females with a mean age of 49.8 years [13]. Tumor markers including CEA, CA19-9, and alpha-fetoprotein are usually normal; even elevated values are not sufficient for diagnosis of PHNET; furthermore, imaging studies usually reveal nonspecific hypervascular hepatic mass [12]. Therefore, the diagnosis of PHNET is confirmed by a combination of radiological findings and IHC stainings, as well as the exclusion of an extrahepatic primary lesion [14]. Serum CgA, a hydrophilic glycoprotein, is a useful marker with a sensitivity of 85.5% and specificity of 98.5% in follow-up of all NETs [15]. The prognosis of surgically resectable cases of primary hepatic neuroendocrine carcinoma (PHNEC) is favorable [16]. Zhang et al. in 58 cases of PHNEC reported that the 5-year survival rate and mean survival were 80% and 148 months, respectively [17]. Regarding normal radiological findings and the normal value of serum CgA, PHNET or metastatic liver NET could not contribute to the significant increase in liver enzymes and subsequently chronic liver disease in our patient.

The last scenario is reactive neuroendocrine differentiation of cholangiocytes after cholestatic liver injury. The epithelial cell lining of intra- and extrahepatic bile ducts i.e., cholangiocytes, participate in bile formation via secretion of water, bicarbonate, and chloride ion. In cholangiopathies including primary biliary cholangitis or primary sclerosing cholangitis, these cells are pivotal, revealing various specific reactions including non-neoplastic proliferation, epithelial-to-mesenchymal transition, and achieving neuroendocrine phenotype [15]. These activated proliferating cholangiocytes may achieve new phenotypes and generate different soluble mediators to regulate its proliferation as well as survival, apoptosis, and function of parenchymal and mesenchymal liver cells and even elements of the immune system in an autocrine/paracrine manner. Hence, this component not only plays role in the development and progression of liver damage but also in repair mechanisms in the course of chronic liver disease [18]. Likewise, in hepatocyte damage, cholangiocytes cooperate in liver regeneration, secreting several substances including cytokines, growth factors, neuropeptides, and hormones. We emphasized that in the presence of neuroendocrine-like cells in liver biopsy in a patient with chronic liver diseases, after excluding NET using biochemical and radiological modalities, the ability of hepatic cholangiocytes to achieve neuroendocrine phenotype mimicking NET in liver biopsy may be considered [19].

The article "Diagnostic dilemma in a patient with history of medullary thyroid carcinoma and abnormal serum liver enzymes; a case report with six years follow up" was published in 2023. Journal: BMC Endocr Disord.

In conclusion, we reported a case of MTC with a highly elevated serum Ctn level at presentation, being in remission both clinically and para-clinically after total thyroidectomy for more than 6 years. During the patient follow-up, due to progressive rising levels of liver enzymes with a predominantly cholestatic pattern, a liver biopsy was performed that revealed nests of neuroendocrine-like cells in the background of PBC. To justify this medical dilemma, we approached the patient as a multidisciplinary team consisting of a hepatologist, oncologist, radiologist, and pathologist. Considering normal tumor biomarkers and unremarkable imaging, metastatic MTC, as well as PHNET, was ruled out and our findings herald acquiring neuroendocrine phenotype by proliferating cholangiocytes. In this case, we highlighted the importance of a multidisciplinary team approach consist of healthcare professionals from different fields to determine the diagnosis and treatment plan in patients with an unusual manifestation of disease. As limitation, we did not perform the calcium-loaded calcitonin test in the management of this patient. However, the significant decrement of serum calcitonin level in immediate post-operative state as well as nearly undetectable levels of serum calcitonin during the 6-year follow-up, make MTC recurrence as an unlikely condition. However, due to a significant decrease in serum calcitonin level immediately after surgery and an undetectable level of it during the 6-year follow-up, recurrence of medullary thyroid cancer is very unlikely.

## Data Availability

Data are available from the corresponding author on reasonable request.

The article "Diagnostic dilemma in a patient with history of medullary thyroid carcinoma and abnormal serum liver enzymes; a case report with six years follow up" was published in 2023. Journal: BMC Endocr Disord.

## Abbreviations

ALP: Alkaline phosphatase
ATA: American thyroid association
CEA: Carcinoembryonic antigen
CgA: Chromogranin A
CT: Computed tomography
Ctn: Calcitonin
EUS: Endoscopic ultrasound
FNA: Fine needle aspiration
GGT: Gamma-glutamyl transferase
IHC: Immunohistochemical
MTC: Medullary thyroid carcinoma
NET: Neuroendocrine tumor
PBC: Primary biliary cholangitis
PET: Positron emission tomography
PHNET: Primary hepatic neuroendocrine tumor
RET: Rearranged during transfection
Tg: Thyroglobulin
